# Reduction of WDR81 impairs autophagic clearance of aggregated proteins and cell viability in neurodegenerative phenotypes

**DOI:** 10.1371/journal.pgen.1009415

**Published:** 2021-03-17

**Authors:** Xuezhao Liu, Limin Yin, Tianyou Li, Lingxi Lin, Jie Zhang, Yang Li

**Affiliations:** 1 Department of Pharmacology, School of Basic Medical Science, Fudan University, Shanghai, China; 2 Division of Experimental Hematology and Cancer Biology, Department of Pediatrics, Brain Tumor Center, Cincinnati Children’s Hospital Medical Center, Cincinnati, United States of America; 3 Shanghai Key Laboratory of Bioactive Small Molecules, Fudan University, Shanghai, China; Stanford University School of Medicine, UNITED STATES

## Abstract

Neurodegenerative diseases are characterized by neuron loss and accumulation of undegraded protein aggregates. These phenotypes are partially due to defective protein degradation in neuronal cells. Autophagic clearance of aggregated proteins is critical to protein quality control, but the underlying mechanisms are still poorly understood. Here we report the essential role of WDR81 in autophagic clearance of protein aggregates in models of Huntington’s disease (HD), Parkinson’s disease (PD) and Alzheimer’s disease (AD). In hippocampus and cortex of patients with HD, PD and AD, protein level of endogenous WDR81 is decreased but autophagic receptor p62 accumulates significantly. WDR81 facilitates the recruitment of autophagic proteins onto Htt polyQ aggregates and promotes autophagic clearance of Htt polyQ subsequently. The BEACH and MFS domains of WDR81 are sufficient for its recruitment onto Htt polyQ aggregates, and its WD40 repeats are essential for WDR81 interaction with covalent bound ATG5-ATG12. Reduction of WDR81 impairs the viability of mouse primary neurons, while overexpression of WDR81 restores the viability of fibroblasts from HD patients. Notably, in *Caenorhabditis elegans*, deletion of the WDR81 homolog (SORF-2) causes accumulation of p62 bodies and exacerbates neuron loss induced by overexpressed α-synuclein. As expected, overexpression of SORF-2 or human WDR81 restores neuron viability in worms. These results demonstrate that WDR81 has crucial evolutionarily conserved roles in autophagic clearance of protein aggregates and maintenance of cell viability under pathological conditions, and its reduction provides mechanistic insights into the pathogenesis of HD, PD, AD and brain disorders related to WDR81 mutations.

## Author summary

In recent years, a group of clinical studies reported that mutations of WDR81 are related to pathogenesis of human brain disorders. However, the underlying mechanisms of pathogenesis are still unknown. In this study, WDR81 promotes the autophagic clearance of protein aggregates via facilitating the recruitment of autophagic proteins onto protein aggregates. The BEACH and MFS domains of WDR81 are sufficient for its recruitment onto Htt polyQ aggregates, and its WD40 repeats are essential for WDR81 interaction with covalent bound ATG5-ATG12. In hippocampus and cortex of patients with HD, PD and AD, protein level of WDR81 is decreased significantly. Reduction of WDR81 impairs the viability of mouse primary neurons, while overexpression of WDR81 restores the viability of fibroblasts from HD patients.

## Introduction

Neurodegenerative diseases, including HD, PD and AD, are characterized by damage to the brain structure, neuron loss and massive aggregation of undegraded proteins. During the pathogenesis of HD, PD and AD, protein aggregation in the brain becomes more and more severe, which is partially due to defective protein degradation in neuronal cells [1,2]. Autophagy is one of the major machineries for protein quality control. Thus, it is important to understand the regulatory mechanisms of autophagy to maintain the protein quality control.

Autophagy is a lysosome-dependent degradation system required for maintenance of cellular energy and nutrition supply. Defective autophagy/lysosome is implicated in numerous pathological conditions [3–5], and enhanced autophagy and lysosome biogenesis relieve symptoms of neurodegenerative and metabolic disorders [6–8]. Briefly, autophagy initiates with the formation of autophagosomes that enclose cytoplasmic contents, followed by autophagosome-lysosome fusion and cargo degradation in autolysosomes [9–11]. The biogenesis of autophagosomes begins with the induction of phagophores in the cytoplasm in response to a variety of signals, which are sensed and mediated by mTOR and the ULK1/2-ATG13-FIP200 complex in mammals. The Beclin1-VPS34-ATG14L complex generates phosphatidylinositol 3-phosphate (PI3P), which is required for phagophore nucleation. Following that, the elongation of phagophores is regulated by two ubiquitin-like conjugation processes: the first conjugates ATG5 to ATG12, and the second conjugates the microtubule-associated protein 1 light chain 3 (MAP-LC3 or LC3/Atg8) to phosphatidylethanolamine (PE) to form LC3-II, enabling expansion and enclosure of autophagosomal membranes. The completed double-membrane autophagosomes are then trafficked to fuse with lysosomes where their contents are digested [9,10].

During autophagic processes, adaptor proteins participate in recruitment of downstream autophagic proteins [12–15], including WDR81, ALFY, NBR1 and NDP52. WDR81 contains a BEACH (beige and Chediak-Higashi) domain, a MFS (major facilitator superfamily) domain, and six WD40 repeats [16]. Since it has transmembrane domains, WDR81 locates on the membranes of endosomes/lysosomes and autophagosomes to regulate endosome trafficking and autophagy [14,17,18]. Previously, we demonstrated that WDR81 recognizes ubiquitinated proteins (Ub-proteins) and promotes their autophagic clearance under physiological conditions [14]. In recent years, a group of clinical studies reported that mutations of WDR81 are related to pathogenesis of human brain disorders. A missense mutation of WDR81, p.Pro856Lys, was identified in the affected members of a family with CAMRQ2 syndrome (cerebellar ataxia, mental retardation, and dysequilibrium syndrome-2) in Turkey [19]. Furthermore, two new mutations of WDR81 (p.Gln1096* and p.Gly282Glu) have been reported in two independent families with congenital hydrocephalus and cerebellar malformation [20], and one new mutation (p.Arg1333*) was reported in a case with intellectual disability and sensorineural hearing loss [21]. In addition, several WDR81 mutations, including p.Tyr453*, p.His528Tyr, p.Gly579Arg, p.Gln628*, and p.Pro1238Arg, have been identified in patients with microcephaly and extreme impairment of neurological development [22, 23]. However, the mechanisms linking WDR81 mutations and brain disorders are still poorly understood.

Therefore, we tested whether reduction of WDR81 resulted in dysfunctional autophagy and impaired viability in neural cells under pathological conditions. In the present study, we found that protein level of WDR81 was decreased significantly in brains of patients with HD, PD and AD. We also investigated the evolutionarily conserved roles of WDR81 in autophagic clearance of protein aggregates in both cellular and animal models. Overexpression of WDR81 improved cell viability under proteotoxic stress, whereas loss of WDR81 significantly aggravated neuron loss. These findings establish that WDR81 functions as a crucial regulator in autophagic clearance of protein aggregates, which provides valuable insights into pathogenesis of human disorders related to WDR81 mutations and its dysfunction.

## Results

### Decreased WDR81 and accumulated p62 in brains of patients with HD, PD and AD

In a previous study, we demonstrated that WDR81 plays a crucial role in autophagic clearance of Ub-proteins under physiological conditions [14]. Based on evidence that WDR81 mutations are related to severe brain disorders in human [22,23], we wanted to dissect the roles of WDR81 under pathological conditions, especially in neurodegenerative diseases. Firstly, we examined the protein level of endogenous WDR81 in the brains of control individuals (Ctrls) and patients with HD, PD and AD (S1 Table). Notably, protein level of endogenous WDR81 was decreased significantly in hippocampus (Fig 1A, 1B and 1C) and cortex of frontal lobe (Fig 1A, 1D and 1E) of indicated patients compared with Ctrls. In brain samples of Ctrls, we observed that endogenous WDR81 localized in cytosol of neuronal cells (Fig 1A). However, in brain samples of patients, much less endogenous WDR81 was detected in cytosol of cells (Fig 1A). And percentage of WDR81-positive cells was significantly decreased in HD, PD and AD patients compared with Ctrls (Fig 1F 1G and 1H). Secondly, we also found that autophagic receptor p62 was accumulated significantly in both hippocampus and cortex of indicated patients compared with Ctrls, suggesting that autophagy was dysfunctional in HD, PD and AD patients (Figs 1I–1L and S1). These results suggested to us that decreased level of WDR81 protein may result in p62 accumulation and autophagy dysfunction, which in turn might exacerbate the pathogenesis of HD, PD and AD.

**Fig 1:** WDR81 is decreased in brains of patients with indicated neurodegenerative diseases compared with brains of control individuals. (A) Representative images of IHC staining of endogenous WDR81 proteins in hippocampus and cortex of brains from Ctrls and patients with AD, HD and PD. Boxed regions are magnified to show change of endogenous WDR81 in cytosol of cells. (B) Quantification of endogenous WDR81 in hippocampus of Ctrls and patients with indicated neurodegenerative diseases separately. 220 cells in 10 fields of each sample were measured. (C) Quantification of endogenous WDR81 in hippocampus of 12 Ctrls and 12 patients with indicated neurodegenerative diseases together. 220 cells in 10 fields of each sample were measured. (D) Quantification of endogenous WDR81 in cortex of frontal lobe from Ctrls and patients with indicated neurodegenerative diseases separately. 260 cells in 10 fields of each sample were measured. (E) Quantification of endogenous WDR81 in cortex of frontal lobe from 12 Ctrls and 12 patients with indicated neurodegenerative diseases together. 260 cells in 10 fields of each sample were measured. (F and G) Ratio of WDR81-positive cells in the sections of hippocampus and cortex of frontal lobe from Ctrls and indicated patients separately. 300 cells in 10 fields of each sample were measured. (H) Ratio of WDR81-positive cells in the sections of hippocampus and cortex of frontal lobe from 12 Ctrls and 12 indicated patients together. 300 cells in 10 fields of each sample were measured. (I) Representative images of IHC staining of endogenous p62 in hippocampus and cortex of brains from Ctrls and patients with HD. (J) Quantification of endogenous p62 in hippocampus of Ctrls and patients with indicated neurodegenerative diseases separately. 280 cells in 10 fields of each sample were measured. (K) Quantification of endogenous p62 in cortex of frontal lobe from Ctrls and patients with indicated neurodegenerative diseases separately. 280 cells in 10 fields of each sample were measured. (L) Quantification of endogenous p62 in the sections of hippocampus and cortex of frontal lobe from 12 Ctrls and 12 indicated patients together. 280 cells in 10 fields of each sample were measured. Scale bars represent 50 μm in all panels. Brain samples from 12 Ctrls and 12 patients with indicated neurodegenerative diseases (AD, n = 4; HD, n = 3; PD, n = 5) were obtained from the Chinese Brain Bank of Zhejiang University (S1 Table). For quantifications, data were calculated by software Image J and analyzed using ANOVA or *t*-test (Prism). ** P <0.01, *** P <0.001.

### WDR81 facilitates recruitment of p62, but not ATG5-ATG12, onto Htt polyQ aggregates

Usually, autophagic adaptor proteins were increased due to the compensation effect under proteotoxic stress in neurodegenerative phenotypes. However, in this study we observed that protein level of WDR81 was decreased significantly in patients’ brains. Consistently with that, we also found that mRNA and protein level of endogenous WDR81 was decreased in mouse brains along with the age growth (Fig 2A and 2B). These results raised our hypothesis that decreased WDR81 impaired selective autophagy, which in turn aggravated the accumulation of protein aggregates and pathogenesis of neurodegenerative diseases. To further investigate the roles of WDR81 in selective autophagy in HD, we examined the recruitment of endogenous WDR81 in HeLa cells stably expressing Htt97Q-EGFP, a mutant Huntingtin protein (Htt) which harbors an expanded polyglutamine (polyQ) repeat and forms Htt polyQ aggregates [12, 24–27]. In normal conditions, WDR81 localizes on the membranes of endosomes [17]. After doxycycline (DOX) treatment, which induced the expression of Htt97Q-EGFP and formation of Htt polyQ aggregates within cells, endogenous WDR81 was recruited onto Htt97Q-EGFP aggregates (Fig 2C and 2D).

**Fig 2:** WDR81 facilitates the recruitment of p62 onto Htt97Q-EGFP aggregates. mRNA level of WDR81 was decreased in the brains of male wild-type mice with the growth of age (n = 20 in each group). Protein level of WDR81 was decreased in the brains of male wild-type mice with the growth of age (n = 3 in each group). (C and D) DOX-induced Htt97Q-EGFP aggregates recruited endogenous WDR81 in HeLa cells (C). After doxycycline (DOX, 1 μg/ml) treatment, HeLa cells stably expressed Tet-on Htt97Q-EGFP. Time-course analysis of WDR81 recruitment onto Htt97Q-EGFP aggregates (D). 200 cells were analyzed for the recruitment. White dotted lines are the outlines of cells. (E and F) Recruitment of endogenous autophagic proteins onto Htt97Q-EGFP aggregates after knockdown of WDR81. Insets show the signals from Htt97Q-EGFP (green) and endogenous autophagic proteins (red) in the aggregates indicated by the white arrows in the main images (left panel). Statistical analysis of the percentage of polyQ foci positive for each indicated autophagic protein (right panel). 220 cells were analyzed for the colocalization in each group. (G) Statistical analysis of the percentage of polyQ foci positive for each indicated autophagic protein in WDR81 KO cells. 210 cells were analyzed for the colocalization in each group. (H and I) Recruitment of endogenous WDR81 onto Htt97Q-EGFP aggregates after knockdown of indicated autophagic proteins. HeLa cells stably expressing Htt97Q-EGFP were transfected twice at an interval of 24 h with siRNAs for indicated autophagic proteins. 12 h after the second siRNA transfection, DOX was administrated into medium to induce Htt97Q-EGFP expression (left panel). Statistical analysis of the percentage of polyQ foci positive for endogenous WDR81 (right panel). 240 cells were analyzed for the colocalization in each group. (J and K) Recruitment of endogenous WDR81 onto Htt97Q-EGFP aggregates in WT or ATG5-/- MEFs. For quantifications, means±SEM were derived from three independent experiments and analyzed using *t*-test or ANOVA. ** P <0.01. *** P <0.001. NS, not significant.

Next, we examined the effect of WDR81 on the recruitment of autophagic proteins onto polyQ aggregates. Knockdown of WDR81 (siWDR81) significantly reduced the recruitment of endogenous autophagic receptor p62 onto Htt97Q-EGFP aggregates (Figs 2E, 2F and S2A), whereas the endogenous ATG12 was still recruited onto Htt polyQ aggregates (Fig 2E and 2F). Consistently, WDR81 deficiency attenuated the recruitment of endogenous p62, but not endogenous ATG12, onto polyQ foci (Fig 2G).

Then, we examined the recruitment of endogenous WDR81 onto Htt97Q-EGFP aggregates after knockdown of ATG5, ATG12 or p62, using specific small interfering RNAs (siRNAs) separately (S2B and S2C Fig). Compared with cells of control group (siCtrl), knockdown of ATG12 (siATG12) or ATG5 (siATG5) abolished the recruitment of endogenous WDR81 onto Htt97Q-EGFP aggregates (Fig 2H and 2I). However, the recruitment of WDR81 was not significantly changed by knockdown of autophagic receptor p62 (Fig 2H and 2I). We also examined WDR81 recruitment onto polyQ foci in WT or ATG5 KO MEFs. Compared with WDR81 in WT MEFs, much less WDR81 was recruited onto Htt polyQ foci in ATG5 KO MEFs (Fig 2J and 2K). Thus, these results demonstrated that WDR81 executed its function as an adaptor protein acting downstream of covalent bound ATG5-ATG12 and upstream of p62 during the autophagic clearance of Htt polyQ aggregates.

### Decreased WDR81 impairs the autophagic clearance of Htt polyQ aggregates

Furthermore, we found that decreased WDR81 resulted in significant accumulation of Htt97Q-EGFP aggregates (Fig 3A and 3B). Consistently, we performed TEM (transmission electron microscopy) assay and found that the number of autophagosomes with undegradated cargoes was significantly increased in WDR81 KO cells compared with WT cells under proteotoxic stress induced by Htt97Q aggregates (S3 Fig). To accurately quantify the diminished recruitment of p62 and accumulation of Htt polyQ aggregates, we administrated DOX to induce expression of Htt97Q-EGFP in stable cell line, and then resuspended and divided these cells into indicated groups followed by RNAi or inhibitor treatments. Subsequently, we performed western blotting to examine levels of polyQ aggregates and did statistics. Firstly, after immunoprecipitation, siWDR81 treatment significantly reduced the association of Htt97Q-EGFP aggregates with endogenous p62 and LC3-II, but not with covalent bound ATG5-ATG12 (Fig 3C and 3D). Secondly, we observed that overexpression of Flag-tagged WDR81 promoted clearance of Htt97Q-EGFP aggregates and autophagic proteins (Fig 3E–3I). And this effect of WDR81 was dependent on lysosome and autophagy activity, since v-ATPase inhibitor Bafilomycin A1 (BafA1) or siATG5 treatments reversed overexpressed WDR81-promoted clearance of polyQ aggregates and autophagic proteins significantly (Fig 3E–3M). Thirdly, we performed overexpression of Flag-tagged WDR81 in WDR81 KO cells expressing Htt97Q-EGFP. We found that overexpression of WDR81 enhanced the recruitment of autophagic receptor p62, but not ATG12 (S4 Fig). Taken together, these results demonstrated that WDR81 promoted autophagic clearance of Htt polyQ aggregates.

**Fig 3:** WDR81 promotes the autophagic clearance of Htt97Q-EGFP aggregates. (A and B) Number of Htt97Q-EGFP inclusions without (siCtrl) or with knockdown of WDR81 (siWDR81) in HeLa cells stably expressing Htt97Q-EGFP. 12 h after the second siRNA transfection, DOX was administrated into medium to induce Htt97Q-EGFP expression. 200 cells in 10 fields of each sample were measured. White dotted lines are the outlines of cells. (C and D) Knockdown of WDR81 reduces association between Htt97Q-EGFP and endogenous p62 and LC3-II, but not covalent bound ATG5-ATG12. Representative images of immunoprecipitation of Htt97Q-EGFP and indicated proteins were shown in the upper panel. Statistical analysis of the association between Htt97Q-EGFP and indicated proteins was shown in the bottom panel. (E-I) WDR81-mediated clearance of Htt97Q-EGFP was dependent on lysosome activity. DOX was added to induce Htt97Q-EGFP expression. 12 h later, Flag-WDR81 (1.5 μg) was transfected into cells. After 12 h, v-ATPase inhibitor, BafA1 (0.4 μM) was added into medium to block capacity of lysosomal degradation. Statistical analysis of clearance of Htt97Q-EGFP and autophagic proteins was shown in the bottom panels. (J-M) WDR81-mediated clearance of Htt97Q-EGFP was dependent on ATG5-mediated autophagy. HeLa cells stably expressing Htt97Q-EGFP were transfected twice at an interval of 24 h without or with siATG5. 12 h after the second siRNA transfection, DOX was administrated into medium to induce Htt97Q-EGFP expression. 12 h later, Flag-WDR81 (1.5 μg) was transfected into cells to promote clearance of Htt97Q-EGFP. Statistical analysis of clearance of Htt97Q-EGFP and autophagic proteins was shown in the right panels. Scale bars represent 10 μm in all panels. For quantifications, means±SEM were derived from three independent experiments and analyzed using ANOVA. * P <0.05. ** P <0.01. *** P <0.001. NS, not significant.

### The BEACH and MFS domains are important to WDR81 recruitment onto Htt polyQ aggregates

Human WDR81 has three major domains, including BEACH domain, MFS domain, and WD40 repeats (Fig 4A). We made truncations of WDR81 to determine which domains are sufficient for recruitment of WDR81 onto Htt polyQ aggregates. Transiently overexpressed EGFP-tagged WDR81 truncations were evenly distributed in cytosol in HeLa cells without expressing Htt polyQ aggregates (S5 Fig). While in HeLa cells with overexpression of Htt97Q-RFP, WDR81(1–650), WDR81(731–1437) and WDR81(1–1636) were normally recruited onto Htt97Q-RFP aggregates similarly as the full-length WDR81 (Fig 4B and 4C). However, WDR81(1637–1940) showed a significant reduction of the WDR81 recruitment onto Htt97Q-RFP aggregates (Fig 4B and 4C). Furthermore, we also made truncations of WDR81 without the BEACH domain or the MFS domain. And we found that lack of BEACH or MFS domain resulted in the significant reduction of WDR81 recruitment onto polyQ aggregates (Fig 4D and 4E). These results demonstrated that the BEACH and MFS domains, but not the WD40 repeats, are sufficient for the recruitment of WDR81 onto Htt97Q aggregates.

**Fig 4:** The BEACH and MFS domains are sufficient for WDR81 recruitment onto Htt97Q aggregates. (A) Schematic representations of full-length and truncations of human WDR81 protein analyzed in present study. Indicated mutations of WDR81 are shown in the BEACH and MFS domains. (B and C) Recruitment of indicated truncations of EGFP-WDR81 onto Htt97Q-RFP aggregates (left panel). Plasmids of Htt97Q-RFP and EGFP-WDR81 were co-transfected into HeLa cells at the same time. 48 h later, recruitment of indicated proteins was observed by fluorescent microscopy. Quantification of the percentage of polyQ foci positive for indicated EGFP-WDR81 truncations is shown in the right panel (C). 200 cells were analyzed for the recruitment in each group. (D and E) Recruitment of mCh-WDR81 without BEACH domain (651–1940) or mCh-WDR81 without MFS domain onto Htt97Q-EGFP aggregates (upper panel). Plasmids of Htt97Q-EGFP and mCh-WDR81 were co-transfected into HeLa cells at the same time. 48 h later, recruitment of indicated proteins was observed by fluorescent microscopy. Quantification of the percentage of polyQ foci positive for indicated mCh-WDR81 truncations is shown in the bottom panel (E). 215 cells were analyzed for the recruitment in each group. (F and G) Colocalization of Htt97Q-EGFP foci with wild-type (WT) or mutant mCherry-WDR81 (mCh-WDR81). Quantification of the percentage of polyQ foci positive for indicated WT or mutant mCh-WDR81 is shown in the bottom panel (G). 210 cells were analyzed for the recruitment in each group. (H-L) Immunoblotting analysis of Htt97Q-EGFP and autophagic proteins without or with overexpression of WT or mutant mCh-WDR81 in WDR81 KO HeLa cells. Fold changes of Htt97Q-EGFP (I) and autophagic proteins (J-L) were normalized to control (vector). Scale bars represent 10 μm in all panels. For quantifications, means±SEM were derived from three independent experiments and analyzed using *t*-tests or ANOVA. ** P <0.01. ***P <0.001.

According to clinical studies, nearly 14 mutants of WDR81 have been reported in human patients with severe neuronal disorders [22, 23]. Therefore, we tested whether autophagic function of WDR81 was impaired by these mutations. Firstly, the WDR81(P856L) mutation locates in the MFS domain and was identified in a family with CAMRQ2 syndrome (Fig 4A) [19]. Compared with mCh-WDR81(WT), mCh-WDR81(P856L) was much less effectively recruited by Htt97Q-RFP foci (Fig 4F and 4G). Recently, clinical case reports showed that patients with congenital brain malformations had mutations of WDR81, including WDR81(H528Y) and WDR81(P1238R) [23], which locate in BEACH and MFS domains of WDR81, respectively (Fig 4A). Similar to WDR81(P856L), overexpressed WDR81(H528Y) and WDR81(P1238R) were also much less effectively recruited onto polyQ foci in WDR81-deficient cells (Fig 4F and 4G).

Secondly, we further performed western blotting to quantify the clearance of Htt97Q aggregates after overexpressing wild-type WDR81 or above mutant WDR81. Consistently, overexpression of wild-type WDR81 promoted the degradation of Htt97Q (Fig 4H and 4I). However, overexpression of mutant WDR81(P856L), which failed to be recruited by Htt97Q aggregates and further aggravated the accumulation of Htt97Q aggregates (Fig 4H and 4I). Similar to WDR81(P856L), overexpression of WDR81(H528Y) or WDR81(P1238R) also blocked the clearance of Htt97Q aggregates (Fig 4H and 4I). Moreover, overexpression of above mutant WDR81 resulted in significant accumulation of autophagic proteins compared with cells overexpressing wild-type WDR81 (Fig 4H–4L).

Thirdly, as the biological consequence of WDR81 recruitment and polyQ degradation, overexpression of WDR81(WT) restored cell viability impaired by Htt97Q induction in WDR81-deficient cells (S6B Fig). To test the defective function of WDR81 mutations, we performed transfection of mCh-tagged WDR81(H528Y), WDR81(P856L), and WDR81(P1238R) in WDR81-deficient cells, respectively. Without the proteotoxic stress, these WDR81 mutations did not significantly change the cell viability (S6A Fig). However, after Htt97Q-EGFP induction in WDR81 KO cells, overexpression of the mutant WDR81 did not restored the cell viability (S6B Fig). Taken together, these results demonstrated that recruitment of WDR81 onto Htt polyQ aggregates promoted clearance of Htt polyQ aggregates and restored cell viability, and this cellular process was dependent on the BEACH and MFS domains of WDR81.

### WD40 repeats are important to WDR81 interaction with covalent bound ATG5-ATG12

We found that knockdown of ATG12 and ATG5 deficiency significantly blocked WDR81 recruitment onto Htt polyQ (Fig 2H–2K), and siATG5 reversed overexpressed WDR81-mediated the autophagic clearance of polyQ aggregates (Fig 3J and 3K). Given these results, we want to characterize the interaction of WDR81 with ATG5 and ATG12 using co-IP assays. After transfection, mCherry-tagged ATG5 and ATG12 were overexpressed and formed a covalent bond within cells. Then, they were efficiently co-immunoprecipitated with Flag-WDR81 (S7A Fig). In addition, ATG5 and ATG12 preferentially bound to the C-terminal WD40 repeats of WDR81(1637–1940) (S7B Fig), but not the N-terminal of WDR81(1–650) (S7C Fig), indicating that WDR81 interacted with ATG5 and ATG12 through its WD40 repeats. Therefore, these results suggested that eventhough Htt polyQ aggregates recruited WDR81 through its BEACH and MFS domains, but the interaction of ATG5-ATG12 with WDR81 through its WD40 repeats could be important for WDR81 stably attaching with polyQ aggregates after the recruitment. That explained the reason why knockdown of ATG12 and ATG5 deficiency significantly decreased the WDR81 recruitment onto Htt polyQ aggregates.

### The functions of WDR81/SORF-2 in autophagy are evolutionarily conserved

Since human WDR81 and *C*. *elegans* SORF-2 share high sequence homology in BEACH domain and WD40 repeats, we examined whether they have conserved functions in the autophagic clearance of aggregated proteins. Firstly, we introduced into *sorf-2(tm5210)* deletion mutants an integrated array, *bpIs267*, which expresses GFP-tagged SQSTM-1/p62 (SQSTM-1::GFP) in hypodermal cells [28]. Whereas no obvious focal structures were found in hypodermis of wild-type (N2) animals, a large number of SQSTM-1::GFP foci were observed in hypodermis of *sorf-2(tm5210)* deletion mutants (Fig 5A and 5B), indicating that SORF-2 was required for eliminating SQSTM-1/p62 bodies.

**Fig 5:** WDR81 has an evolutionarily conserved effect on autophagic clearance of protein aggregates and maintenance of cell viability. (A) *C*. *elegans sorf-2(tm5210)* mutants accumulate p62/SQSTM-1::GFP foci in hypodermal cells, which is rescued by expression of either *C*. *elegans sorf-2* or human *WDR81* driven by a hypodermal cell-specific promoter (P_*Y37A1B*.*5*_). (B) Quantification of SQSTM-1::GFP foci in wild-type, *sorf-2(tm5210)*, and *sorf-2(tm5210)* animals carrying transgenes expressing *sorf-2* or *WDR81*. The indicated numbers of animals from each genotype were analyzed for hypodermal SQSTM-1::GFP intensity (arbitrary units, AU); 3 independent lines are shown for *sorf-2* or *WDR81* transgenes. *, compared with WT group. #, compared with *sorf-2(tm5210)* group. (C and D) GFP-positive DA neuron loss induced by α-synuclein is exacerbated in *sorf-2(tm5210)* mutants. Representative images of a *baIn1* (*P*_*dat-1*_:: α-synuclein+ *P*_*dat-1*_:: GFP) animal with all 6 DA neurons (white arrows) and a *baIn1* animal with 2 DA neurons are shown in the left panels. Quantifications of DA neuron loss in *baIn1* and *sorf-2(tm5210); baIn1* animals are shown in the right panel (D). Data were derived from 3 independent quantifications in which ≥40 animals of each genotype were scored for DA neurons at every time point. (E) Overexpression of *sorf-2* or *WDR81* rescues GFP-positive DA neuron loss induced by α-synuclein in *sorf-2(tm5210)* mutants. ≥50 animals were scored for DA neurons in each of 3 independent transgenic lines expressing *sorf-2* or *WDR81* driven by a neuron-specific promoter (P_*dat-1*_). Data presented are from animals at the age of 4 or 6 days post the L4 molt. (F-J) Knockdown of WDR81 resulted in accumulation of Htt97Q aggregates and endogenous autophagic proteins in mouse primary neurons. Primary neurons were isolated from cortex of C57/B6 mouse brains. Representative images were shown from 3 independent experiments (F). Statistical analysis was performed to test fold changes of indicated proteins (G-J). (K) Viability of mouse primary cortex neurons transiently expressing Htt97Q-EGFP without or with siWDR81 treatment. (L)Viability of mouse primary cortex neurons transiently expressing Htt97Q-EGFP without or with overexpression of wild-type WDR81. (M) Viability of Htt68-containing fibroblasts from HD patients without or with siWDR81 treatment. (N) Viability of fibroblasts from two HD patients with two different polyQ expansions (Htt47Q and Htt68Q), was restored by overexpression of wild-type full-length WDR81. Scale bars represent 20 μm in all panels. For quantifications, means±SEM were derived from three independent experiments and analyzed using *t*-test or ANOVA. * P <0.05, ** P <0.01, *** P <0.001.

Secondly, we crossed into *sorf-2(tm5210)* mutants an integrated array (*baIn1*), which ectopically expresses α-synuclein (α-Syn) in 6 GFP-positive dopaminergic (DA) neurons in the head [29]. α-Syn is known to form neuron-toxic aggregates that are removed by macroautophagy [30], whereas its soluble form is eliminated by chaperone-mediated autophagy [31,32]. In wild-type *C*. *elegans* animals, ectopic expression of α-Syn caused loss of GFP-positive DA neurons in an age-dependent manner, which manifested as a progressive age-related decrease in the population of animals possessing all 6 DA neurons (Fig 5C) [29,33]. In *sorf-2(tm5210)* deletion mutants, α-Syn-induced loss of DA neurons was greatly exacerbated, as evidenced by a significant decrease in the population of animals with 6 DA neurons at all age points examined (Fig 5C and 5D). These results suggested that SORF-2 was essential for clearance of the toxic ectopically expressed α-Syn in DA neurons. Taken together, these results indicated that *C*. *elegans* SORF-2 had a similar role to human WDR81 in removing aggregated proteins.

To test if WDR81 functions in an evolutionarily conserved manner in removal of aggregated proteins and maintenance of neuron viability, we used a hypodermis-specific promoter to drive the expression of either *C*. *elegans* SORF-2 or human WDR81 in *sorf-2(tm5210)* mutants and examined the level of SQSTM-1::GFP foci. In all transgenic lines of *sorf-2(tm5210)* expressing either SORF-2 or WDR81, the accumulation of SQSTM-1::GFP foci in hypodermis was ameliorated to an extent similar to that in wild-type animals (Fig 5A and 5B). This indicated that WDR81 replaced SORF-2 in removing protein aggregates in *C*. *elegans*. Likewise, α-Syn-induced GFP-positive DA neuron loss in *sorf-2(tm5210)* mutants was rescued to a level similar to that in wild type by expressing SORF-2 or WDR81 driven by a neuron-specific promoter P_*dat-1*_ (Fig 5E). This provided strong evidence that WDR81 had a conserved function in metazoa in the clearance of aggregated proteins and maintenance of neuron viability.

Moreover, the protective effect of human WDR81 on restoring DA neuron viability in worms strongly suggested to us that WDR81 could maintain neuron viability under proteotoxic stresses. To prove that, firstly we performed transient transfection of Htt97Q-EGFP and the siRNA of WDR81 in primary mouse cortex neurons *in vitro* culture. Then, we performed western blotting and found that siWDR81 treatment aggravated the accumulation of both Htt97Q aggregates and endogenous autophagic proteins (Fig 5F–5J). Meanwhile, reduction of WDR81 aggravated neuron death induced by Htt97Q-mediated proteotoxic stress in cortex neurons (Fig 5K). However, overexpression of WDR81 increase viability of mouse neurons impaired by Htt97Q aggregates (Fig 5L).

Notably, the protective effect of WDR81 under proteotoxic stress was conserved not only in worm and mouse neurons, but also in patients’ fibroblasts. We obtained fibroblasts from control individuals and HD patients with two different polyQ expansions, Htt47Q and Htt68Q [34], respectively. Similarly, reduction of WDR81 aggravated cell death induced by proteotoxic stress in Htt68Q-containing fibroblasts (Fig 5K). Interestingly, fibroblasts from HD patients were more vulnerable compared with Ctrl fibroblasts (Fig 5N), whereas overexpression of WDR81 significantly restored the viability of patients’ fibroblast (Fig 5N). Taken together, these results provided evidence that WDR81 had conserved functions to maintain cell viability under proteotoxic stresses.

## Discussion

In this study, we demonstrate that reduction of WDR81 results in dysfunctional autophagic clearance of protein aggregates and impairs cell viability in neurodegenerative phenotypes. Firstly, we find that patients with HD, PD and AD, have significant reduction of WDR81 and accumulation of p62 in the hippocampus and cortex of brains. Then, we identify that the BEACH and MFS domains of WDR81 are essential for recruitment of WDR81 onto Htt polyQ aggregates. And WD40 repeats of WDR81 are important to its interaction with ATG5-ATG12. Furthermore, WDR81 facilitates the recruitment of its downstream autophagic proteins, and has evolutionarily conserved roles in maintaining the viability of neuronal cells in both worms and mammalian cells. Taken together, our findings demonstrate that WDR81 functions as an adaptor protein to facilitate recruitment of autophagic regulators on protein aggregates, thereby promoting the clearance of aggregates under proteotoxic stresses and pathological conditions (Fig 6).

**Fig 6:** Model of WDR81-mediated autophagic clearance of protein aggregates.

WDR81 is abundantly expressed, especially highly expressed in brains [14]. Our previous study found that conditional KO of WDR81 in mouse neurons results in fetal death and robust accumulation of Ub-proteins in brains under the physiological conditions [14]. Consistently, in this study, we observe that WDR81 is reduced significantly in mouse brains with the growth of age, and its protein level is also decreased significantly in neurodegenerative patients’ brains. Furthermore, we demonstrate that decreased WDR81 impairs selective autophagy for the clearance of protein aggregates, and its reduction also impairs the neuron viability subsequently. Therefore, we conclude that reduction of WDR81 is one of the causes of neurodegenerative pathogenesis in aged human beings.

Consistent with our data, another study also demonstrated that the WDR81(L1349P) mutation results in Purkinje cell degeneration and photoreceptor cell loss in mice [16]. Importantly, a point mutation (P856L) in WDR81 was reported to be associated with human CAMRQ2 syndrome [19]. Several mutations of WDR81 are associated with clinical brain and nervous system phenotypes in human, including cerebellar ataxia, mental retardation, congenital hydrocephalus and impairment of neurological development [22,23]. In our previous work, we reported that WDR81 interacts with p62 and LC3 via its BEACH domain (S2 Table). In present study, we find that WDR81 interacts with ATG5-ATG12 via its WD40 repeats (S2 Table). Besides, BEACH and MFS domains of WDR81 are sufficient for its recruitment onto Htt polyQ aggregates under pathological conditions (S2 Table). Most of WDR81 mutations locate in the BEACH, MFS domains and WD40 repeats of WDR81, which are essential for the recruitment of WDR81 onto protein aggregates and its interaction with autophagic proteins (Fig 4 and S2 Table). We speculate that these mutations, including H528Y, P856L, P1238R and L1349P, may localize in the certain conformational regions, which are crucial to form pocket-like structures for the functions of WDR81 as an adaptor protein. That may be the reason why only a single mutation can diminish WDR81 recruitment and autophagic clearance of protein aggregates (Fig 4). Taken together, these lines of evidence suggest that WDR81 mutations compromise the normal functions of WDR81, thus impairing neuron viability and protein quality control.

Recently, Guo’s group reported that loss of WDR81 in adult neural progenitor cells significantly reduced adult neurogenesis in hippocampus and impaired hippocampus-dependent learning [35]. Thus, this study supports our conclusion that WDR81 reduction is the one of the causes of neurodegenerative disorders. Since we also found WDR81 reduction in hippocampus of patients’ brains, its reduction not only impairs selective autophagy and protein quality control, but also may impair adult neurogenesis and hippocampus-dependent learning and memory, which in turn aggravates the pathogenesis of neurodegeneration.

Our findings that loss of WDR81 function led to accumulation of misfolded proteins, which likely renders the cells sensitive to induction of apoptosis, suggest that WDR81 is relevant to aggregate-associated neuron loss in HD, PD and AD. Consistent with this, α-synuclein-induced DA neuron loss was significantly exacerbated in *C*. *elegans sorf-2/*WDR81 mutants. Since overexpression of human WDR81 can rescue the phenotype of *sorf-2* mutants, the effects of WDR81 on autophagic clearance of protein aggregates and maintenance of neuron viability are evolutionarily conserved.

In addition, given that mutations of other BEACH domain-containing proteins (BDCPs) are reported to be associated with diseases, including Chediak-Higashi syndrome (CHS), defects in the immune system, and autism [36], it will be necessary to explore whether the functions of those BDCPs are related to the regulation of autophagy and clearance of intracellular materials.

### Experimental procedures

dx.doi.org/10.17504/protocols.io.brg5m3y6

### Ethics statement

For the animal experiments, all procedures were performed according to protocols approved by Animal Ethics Committees at Fudan University (2018-C001). For the experiments using human samples, all procedures were performed according to protocols approved by Human Ethics Committees at both Fudan University and Zhejiang University (2018-C005). Brain samples from 12 control individuals and 12 patients with indicated neurodegenerative diseases (AD, n = 4; HD, n = 3; PD, n = 5) were obtained from the Chinese Brain Bank of Zhejiang University (S1 Table). The obtained formal consent was written.

### Cell culture, reagents, and transfection

Cells were cultured at 37°C with 5% CO_2_ in Dulbecco’s modified Eagle’s medium (DMEM) supplemented with 10% fetal bovine serum (FBS) (HyClone, Novato, CA), 100 U/ml penicillin and 100 mg/ml streptomycin. Transfections were performed with Lipofectamine 2000 (Invitrogen, Carlsbad, CA) according to the manufacturers’ instructions. MG132 and doxycycline were obtained commercially. Fibroblasts from control individuals and HD patients with the Htt47Q and Htt68Q expansions were obtained from Dr. Boxun Lu’s lab in Fudan University.

In brief, primary cortex neurons were isolated from appropriately timed pregnant female (16.5 days). Using forceps, we isolated cortex from each hemisphere of mouse brains under microscope. Once the cortex regions were isolated, they were cut into approximately 10 smaller pieces for digestion (1 ml prewarmed Trypsin, at 37°C for 20 min). Then serum was added to inactivate trypsin. After aspirating the supernatant, we added 1 ml prewarmed DNase solution for 10 min at 37°C. Then, the cells were dissociated by pipetting up and down, and all supernatant were transferred to new tubes for subsequent centrifugation (800xg for 5 min). We resuspended cell pellet gently and plated them on coated dishes (Poly-D-Lysine, BD, #354210). The neuronal culture medium was changed every 2 days. After about 14 days of neuronal culture, we performed transient transfection of Htt97Q-EGFP (1 μg) or/and siWDR81 (100 pmol, three times at an interval of 24 h) using Lipofectamine MessengerMAX (Thermo Fisher Scientific) as manufacturing introduction.

### Immunostaining and confocal microscopy

Cells grown on coverslips were fixed in 4% paraformaldehyde followed by permeabilization with 0.05% saponin. After extensive washing with phosphate buffered saline (PBS), cells were incubated with primary antibodies in PBS containing 5% BSA at 4°C overnight. Cells were washed extensively again and incubated with secondary antibodies for 1 h at room temperature. Following another round of thorough washing, cells were sealed on slides for microscopy analysis. For live cell imaging, cells were grown in confocal dishes (Glass Bottom Dish, In Vitro Scientific, Sunnyvale, California, USA). Samples were examined with an inverted Olympus FV1000 confocal microscope. Images were analyzed with FV10-ASW 4.0a Viewer.

### Generation of cell lines stably expressing Tet-on Htt97Q-GFP

HeLa cells stably expressing pcDNA6/TR (kindly provided by Dr. Quan Chen) were transfected with pcDNA4-Htt97Q-GFP. 24 h later, cells were subjected to selection for 2–3 weeks in medium supplemented with blasticidin (5 μg/ml) and zeocin (100 μg/ml). Single colonies were picked and propagated further. The expression of Htt97Q-GFP was determined by adding doxycycline (1 μg/ml) and observed by fluorescence microscopy.

### Htt polyQ clearance assay

To assess the effect of siRNA knockdown of WDR81 on clearance of Htt polyQ inclusions, HeLa cells stably expressing Tet-on Htt97Q-EGFP were transfected twice at an interval of 24 h with siRNA oligos against WDR81. 12 h after the second siRNA transfection, Htt97Q-EGFP expression was induced with doxycycline (1 μg/ml). The medium was changed 12 h later to remove the doxycycline and the cells were split into several dishes for the remaining siRNA treatments. Time-course quantification of polyQ foci was performed 12 h after the induction of Htt97Q-EGFP expression. To rescue WDR81 siRNA-induced accumulation of polyQ foci, cells were first treated with control or WDR81 siRNA, then 3 μg of vector expressing siRNA-resistant WDR81 were transfected into the same cells simultaneous with the induction of Htt97Q-EGFP expression by doxycycline. siRNA treatments were performed twice more as above and polyQ foci were scored 48 h post induction of Htt97Q-EGFP expression.

### C. elegans genetics

*C*. *elegans* Bristol strain N2 was used as wild type. *sorf-2(tm5210)* deletion mutants were provided by Dr. Shohei Mitani (Tokyo Women’s Medical University, Japan). The integrated arrays *bpIs267* and *baIn1* were kindly provided by Dr. Hong Zhang (Institute of Biophysics, CAS, China) and Dr. Guy Caldwell (University of Alabama, Tuscaloosa). *C*. *elegans* cultures, genetic crosses, and generation of transgenic animals were performed according to standard procedures (Brenner 1974).

### Human subjects and IHC procedure

Brain samples from 12 control individuals and 12 patients with indicated neurodegenerative diseases (AD, n = 4; HD, n = 3; PD, n = 5) were obtained from the Chinese Brain Bank of Zhejiang University (S1 Table). The samples are paraffin-embedded sections of hippocampus and cortex of frontal lobe. The controls and patients were strictly paired according to parameters including age, gender, reason of death and phase of disease. All procedures were performed according to protocols approved by Human Ethics Committees at both Fudan University and Zhejiang University.

Paraffin-embedded sections were dewaxed, rehydrated, and rinsed in PBS. After being boiled for 15 min in 0.01 mol/liter sodium citrate buffer (pH 6.0), sections were blocked in 5% guinea pig (Gp) or rabbit pre-immune serum in PBS for 1 h at room temperature and then incubated overnight with WDR81 antibody (Gp, 1:200) or p62 antibody (rabbit, 1:1000). Sections were then incubated in horseradish peroxidase-conjugated secondary antibody (1:200) at room temperature for 3 hours. After 4 washes in PBS, 3,3-diaminobenzidine (DAB) was added for 1 min at room temperature. Sections were counterstained with hematoxylin for 2 min. The IHC pictures were obtained by Nikon microscope (Ts2R). Results were calculated by software Image J and NIS-Element, BR. 3.00 (Nikon). For quantification measurements, images were randomly acquired from the hippocampus and cortex of frontal lobe and analyzed by researchers in a double-blind manner.

### Expression vectors

The mammalian, bacterial and *C*. *elegans* expression vectors listed in **S3 Table** were constructed using standard protocols [14].

The vector, pcDNA3.1-Htt97Q-EGFP, was kindly provided by Dr. Xiaojiang Li (Institute of Genetics and Developmental Biology, CAS, China).

### Small interfering RNAs (siRNAs)

The oligos used for siRNA knockdown of WDR81 were as described previously [14]. Other oligos were as follows: p62: 5’-GCATTGAAGTTGATATCGAT-3’[37];

ATG12: 5’-AUGAGCUUCAAUUGCAUCCtt-3’ [38];

Control siRNA: 5’-UUCUCCGAACGUGUCACGUTT-3’.

Cells were transfected with 100 pmol siRNA oligos twice at an interval of 24 h. Cells were subjected to further analysis 24 h after the last transfection. For the transfection of primary neurons, we performed the assay using Lipofectamine MessengerMax reagent (Invitrogen).

### Quantitative reverse transcription–polymerase chain reaction (qPCR)

Total RNA was extracted using Trizol (Invitrogen) and chloroform. 2 μg of RNA was used as template to generate cDNAs using the ImProm-II Reverse Transcription system (Promega, Madison, Wisconsin, USA). qPCR reactions were carried out on an MX3000P system (Agilent Technologies, Santa Clara, CA).

### Antibodies

WDR81 antibodies were generated in guinea pigs and rabbits by injecting purified recombinant GST-WDR81(332–604) and purchased from ABclonal (#A12780). GFP and mCherry antibodies were generated in guinea pigs or rabbits by injecting recombinant proteins. Rabbit polyclonal antibodies to p62 were purchased from Medical & Biological Laboratories (MBL, Nagoya, Japan). Mouse monoclonal antibodies against ATG12 were purchased from MBL. Mouse monoclonal antibodies to β-actin and GFP were purchased from Sigma-Aldrich (St. Louis, MO). HRP-, Cy3-, and FITC-conjugated secondary antibodies were from Jackson ImmunoResearch Laboratories (West Grove, PA).

### Western blotting and immunoprecipitation

To analyze levels of proteins of interest, cells were lysed in ice-cold Triton X-100 buffer (20 mM Tris-HCl, pH7.5, 100 mM NaCl, 1% TritonX-100, 1 mM phenylmethanesulfonyl fluoride (PMSF)) or RIPA buffer (20 mM Tris-HCl pH7.5, 100 mM NaCl, 0.1% SDS, 0.5% Sodium deoxycholate, 1 mM PMSF) containing one Complete Protease Inhibitor Cocktail Tablet (Roche, Basel, Switzerland). Cell lysates were spun down at 12000 rpm for 10 min. 50 g of supernatants were resolved on sodium dodecyl sulfate polyacrylamide gels (SDS-PAGE) and blotted with the indicated antibodies. β-actin was used as the loading control.

To determine the interaction of endogenous WDR81 with autophagy factors or Htt polyQ-associated proteins, HeLa cells with or without Htt97Q-EGFP expression were lysed in ice-cold Triton X-100 buffer containing one Complete Protease Inhibitor Cocktail Tablet (Roche). In the case of Htt97Q-EGFP IP, the cell lysates were cleared by centrifugation at 500xg as described by Filimonenko et al. [12]. Cleared cell lysates were first mixed with antibodies to WDR81 or GFP (~5 μg) for 4 h followed by incubation with protein A agarose beads (10 μl) (GE Healthcare) overnight at 4°C. Analysis of precipitated proteins was performed as above.

### MTT assay for cell viability

The MTT kit was purchased from Promega (#G4002). Cells were cultured in 96-well plates with DMEM containing 10% FBS. After various treatments, 15 μL of dye solution was added into each well. Then the plates were incubated at 37°C for 1.5 hours in a humidified CO_2_ incubator. Stop solution (100 μL) was added into each well, and the absorbance was recorded at 570 nm using plate reader. 630 nm was used as a reference wavelength.

### Transmission electron microscopy

Cells were fixed for 2.5 h at 4°C with 0.1 M PBS containing 2.5% glutaraldehyde. Then, the fixed samples were rinsed with PBS and 1% OsO4 for 0.5 h at 4°C. The samples were rinsed with distilled water and dehydrated by sequential incubation with an acetone series (30%, 50%, 70%, 80%, 90%, 95%, 100%, and 100%, 5 min each). After that, samples were infiltrated with Araldite 502/Embed 812 by gradually increasing the concentration of acetone (25% and 50%, 20 min; 75%, 30 min; 100%, 20 h) and then polymerized at 60°C for 70 h. Embedded samples were sectioned using an UC6 ultramicrotome (Leica Biosystems) equipped with a 45° diamond knife (Diatome) to obtain 70-nm ultrathin sections. The grids were stained at room temperature with 2% aqueous uranyl acetate (10 min) and Reynolds lead citrate (5 min) before imaging. Imaging was performed at 80 kV on a JEM-1400 (JEOL) transmission electron microscope.

### Statistics and reproducibility

Data were analyzed with Prism (GraphPad software). Statistical analyses were performed using *t*-tests or ANOVA. *P<0.05 was considered statistically significant. **P<0.01 was considered significant. ***P<0.001 was considered extremely significant. P>0.05 was considered not significant (NS).

## Supporting information

S1 Fig Representative images of IHC staining of endogenous p62 in hippocampus and cortex of brains from Ctrls and patients with AD or PD. Scale bars represent 50 μm in all panels. Brain samples from 12 Ctrls and 12 patients with indicated neurodegenerative diseases (AD, n = 4; HD, n = 3; PD, n = 5) were obtained from the Chinese Brain Bank of Zhejiang University (S1 Table).
(TIF)

S2 Fig Efficiency of the indicated siRNAs. (A-D) Efficiency of indicated siRNAs. HeLa Cells were transfected with 100 pmol siRNA oligos twice at an interval of 24 hours. Then, mRNA was isolated at 24 h after the last transfection. For quantifications, means±SEM were derived from three independent experiments and analyzed using *t-test*. *** P <0.001.
(TIF)

S3 Fig Representative TEM images of control and KO-81 HeLa cells with Htt97Q-induced proteotoxic stress. (A)Cargo-containing autophagic vesicles (AVs) in cells. Insets in the bottom right corner show magnified views of the yellow arrows-indicating autophagic structures in cells. (B) Quantification of AV numbers observed by TEM. For all quantifications, data (mean ± SEM) were from three independent experiments and analyzed using *t*-test. ***, P < 0.001. Bars, 0.5 μm.
(TIF)

S4 Fig Overexpression of Flag-WDR81 enhanced the recruitment of p62 onto polyQ foci. We performed co-transfection of Htt97Q-EGFP and Flag-WDR81 in WDR81 KO cells. 48 hours later, we did cell fixation and the endogenous staining of autophagic proteins, then the recruitment of endogenous ATG12 (A) or p62 (B) was observed under fluorescent microscopy. For quantifications, data were derived from three independent experiments and analyzed using ANOVA. * P <0.05, ** P <0.01, *** P <0.001.
(TIF)

S5 Fig Full-length or truncated WDR81 did not form aggregates without overexpression of Htt polyQ aggregates. Full-length or truncated EGFP-WDR81 (2 μg) was transfected into HeLa cells. 48 hours later, cells were observed under fluorescent microscopy. Similar as full-length WDR81, indicated truncated EGFP-WDR81 distributed evenly in the cytosol, and none of WDR81 foci were observed.
(TIF)

S6 Fig Overexpression of mutant WDR81 did not restore cell viability impaired by Htt polyQ aggregates in WDR81-deficient cells. (A)Overexpression of WT or mutant WDR81 did not affect cell viability of WDR81 KO cells without expressing Htt polyQ aggregates. (B)Overexpression of WT WDR81, but not mutant WDR81, restored Htt97Q-impaired cell viability in WDR81 KO cells under proteotoxic stress. For quantifications, data were derived from three independent experiments and analyzed using ANOVA. ** P <0.01. NS, not significant.
(TIF)

S7 Fig WD40 repeats of WDR81 are sufficient for its interaction with ATG5-ATG12. (A) Co-IP of Flag-WDR81 with mCh-ATG5 and mCh-ATG12. Flag-WDR81 and the indicated proteins were co-expressed in HEK293 cells. IPs were performed with Flag antibody and precipitated proteins were detected with ATG12 and Flag antibodies. (B and C) Co-IP of mCh-ATG5 and mCh-ATG12 with Flag-WDR81(1637–1940) (B) or Flag-WDR81(1–650) (C). Representative images were shown from three independent experiments.
(TIF)

S1 Table Information about patients with neurodegenerative diseases and paired control individuals. (DOCX)

S2 Table List of WDR81 domains, mutations and related symptoms in patients. In present study, WDR81 recruitment onto Htt polyQ aggregates is dependent on its BEACH and MFS domains. C-terminal WD40 repeats is sufficient for its interaction with ATG5-ATG12. According to our previous study, WDR81 interacts with p62 and LC3 via its BEACH domain. #, the observation was reported in our previous study [14].
(DOCX)

S3 Table The list of expression vectors using in this study. (DOCX)
